# The Nexus between VEGF and NFκB Orchestrates a Hypoxia-Independent Neovasculogenesis

**DOI:** 10.1371/journal.pone.0059021

**Published:** 2013-03-22

**Authors:** Michael DeNiro, Falah H. Al-Mohanna, Osama Alsmadi, Futwan A. Al-Mohanna

**Affiliations:** 1 Research Department, King Khaled Eye Specialist Hospital, Riyadh, Saudi Arabia [Affiliate of the Wilmer Eye Institute/Johns Hopkins Medicine, Baltimore, Maryland, United States of America]; 2 Department of Comparative Medicine, King Faisal Specialist Hospital and Research Centre, Riyadh, Saudi Arabia; 3 Dasman Genome Centre, Dasman Diabetes Institute, Kuwait City, Kuwait; 4 Department of Cell Biology, King Faisal Specialist Hospital and Research Centre, Riyadh, Saudi Arabia; 5 Medical College, Al-Faisal University, Riyadh, Saudi Arabia; INRS, Canada

## Abstract

Nuclear Factor-Kappa B [NFκB] activation triggers the elevation of various pro-angiogenic factors that contribute to the development and progression of diabetic vasculopathies. It has been demonstrated that vascular endothelial growth factor [VEGF] activates NFκB signaling pathway. Under the ischemic microenvironments, hypoxia-inducible factor-1 [HIF-1] upregulates the expression of several proangiogenic mediators, which play crucial roles in ocular pathologies. Whereas YC-1, a soluble guanylyl cyclase [sGC] agonist, inhibits HIF-1 and NFκB signaling pathways in various cell and animal models. Throughout this investigation, we examined the molecular link between VEGF and NFκB under a hypoxia-independent microenvironment in human retinal microvascular endothelial cells [hRMVECs]. Our data indicate that VEGF promoted retinal neovasculogenesis via NFκB activation, enhancement of its DNA-binding activity, and upregulating NFκB/p65, SDF-1, CXCR4, FAK, αVβ3, α5β1, EPO, ET-1, and MMP-9 expression. Conversely, YC-1 impaired the activation of NFκB and its downstream signaling pathways, via attenuating IκB kinase phosphorylation, degradation and activation, and thus suppressing p65 phosphorylation, nuclear translocation, and inhibiting NFκB-DNA binding activity. We report for the first time that the nexus between VEGF and NFκB is implicated in coordinating a scheme that upregulates several pro-angiogenic molecules, which promotes retinal neovasculogenesis. Our data may suggest the potential use of YC-1 to attenuate the deleterious effects that are associated with hypoxia/ischemia-independent retinal vasculopathies.

## Introduction

Angiogenesis is the formation of new blood vessels and capillary beds from existing vessels, which plays a fundamental role in physiological and pathological processes. In physiological conditions, angiogenesis occurs primarily in embryonic development, during tissue and wound repair, and in response to ovulation. However, pathological angiogenesis, or the abnormal rapid proliferation of blood vessels, is implicated in various diseases, including cancer, psoriasis, diabetic retinopathy [DR], and rheumatoid arthritis. Vascular endothelial growth factor [VEGF] is one of the most potent stimuli for new blood vessel growth, and therefore it has emerged as one of the most important growth factors controlling angiogenesis. Under pathological conditions, ischemia/hypoxia develops within the neovascular retina, which in turn increases VEGF levels in part through stabilization of VEGF mRNA [1]. This ischemic effect is mediated primarily by hypoxia inducible factor-1 [HIF-1], which is often considered as the master regulator of angiogenesis under ischemia/hypoxia. Retinal ischemia often precedes the onset of such NV, and the ischemic retina has been identified as a potential source of diffusible angiogenic factors. Retinal neovascularization [NV] is a major cause of the blindness that is associated with ischemic retinal disorders such as DR, retinopathy of prematurity [ROP], and retinal vein occlusion. Despite the prevalence of DR and ROP, an effective treatment for retinal NV remains elusive. Retinal NV is induced by complex interactions among multiple cytokines and adhesion molecules. Several potential inhibitors of retinal NV, including soluble VEGF receptor and antagonists of both αv-integrin and growth hormone have been identified with the use of a highly reproducible model of ischemia-induced retinal NV. Although VEGF is one of the central angiogenic factors induced in the neovascular retina, other growth factors may play crucial roles in the development and progression of retinal NV, many of which are hypoxia-independent. Various therapeutic modalities to inhibit VEGF have shown efficacy in the treatment of ischemia/hypoxia-driven retinal NV [2], [3], [4]. However, hoard evidence indicates that nonischemic microenvironment may also induce retinal NV [5], [6]. Furthermore, it has been demonstrated that in the streptozotocin [STZ]-induced type 1 diabetic rat model [7], [8]; the retinas exhibit most of the pathological features of DR seen in humans, including blood vessel dilation, blood retinal barrier [BRB] breakdown, microaneurysm formation, and intraretinal microvascular abnormalities, which makes this model widely used in studies of the early stages of DR, especially in those examining vascular hyperpermeability in the retina. [9], [10], [11]. In addition, streptozotocin [STZ]-induced diabetes failed to cause any significant increase in either HIF-1α or hypoxia. Interestingly, however, there was even a tendency for hypoxia levels to be decreased [tissue more highly oxygenated] [12].

Nuclear factor kappa-B [NFκB] is a heterodimeric complex of Rel family of proteins that is physically confined to the cytoplasm in unstimulated cells through the binding to inhibitor of κB [IκB] proteins [13]. It has been suggested that VEGF’s activation of NFκB signaling pathway is largely dependent on the cellular context. Both activation [14], [15] and inhibition [16] of NFκB in response to VEGF have been reported. Furthermore, it has been indicated that expression of pro-angiogenic factors, such as; SDF-1, CXCR4, FAK, αVβ3, α5β1, EPO, ET-1, and MMP-9 expression, are mediated by NFκB activation and may contribute to the pathogenesis of intraocular NV in individuals with DR or retinal vein occlusion. YC-1; 3-(5′-Hydroxymethyl-2′-furyl)-1-benzylindazole, has been identified as an sGC, and was shown to increase the intracellular cGMP concentration in platelets [17]. It was further demonstrated that YC-1 may activate the sGC/cGMP/PKG pathway to induce Ras and PI3K/Akt activation, which in turn initiates IKKα/β and NF-κB activation [18]. In addition, it has been established that cyclic GMP regulates NFκB in T Lymphocytes, neuronal cells, cardiomyocytes, endothelial cells, and hepatocytes [19]. These observations suggest that NFκB may represent a suitable target for therapeutic intervention in retinal NV. With the animal model of oxygen-induced retinopathy [OIR], it has been previously shown that nuclear factor KB [NFκB] activation may be important to induce retinal NV. In that model, exposure of neonatal animals to hyperoxic conditions results in extensive obliteration of retinal capillaries. When the animals are returned to room air, the inner retina presumably becomes relatively hypoxic, which results in the activation of NFκB, production of many cytokines, adhesion molecules, and retinal NV. Here, we investigate the molecular nexus between VEGF and NFκB in relation to retinal neovasculogenesis in the absence of the hypoxic microenvironment, and examine the effects of YC-1 on retinal neovasculogenesis in human retinal microvascular endothelial cells [hRMVECs].

## Materials and Methods

### Ethics Statement

All experiments were conducted in compliance with the laws and the regulations of the Kingdom of Saudi Arabia. In addition, all protocols were approved by the Institutional Review Board. This research study was approved by: The King Khaled Eye Specialist Hospital’s Human Ethics Committee & Institutional Review Board [HEC/IRB], Riyadh, Saudi Arabia. The permit number/approval ID is “RP 0630-P”.

### Reagents

YC-1 [Fig. 1A] was purchased from A.G. Scientific [San Diego, CA] and dissolved in sterile DMSO. SN50 [a cell-permeable synthetic peptide, known to inhibit the nuclear translocation of NFκB, and its negative control mutant peptide SN50M were obtained from Calbiochem [San Diego, CA]. TSA™ Kit #4 with Alexa Fluor® 568 tyramide was purchased from Molecular Probes, Inc [Eugene, OR]. Recombinant human VEGF_165_ was purchased from Chemicon [Temecula, CA]. Mouse monoclonal antibody that recognizes the active subunit [12H11] of RELA [NFκB/p65] [MAB3026] was obtained from Millipore [Billerica, MA, USA]. Anti-phospho-IkBα antibody was purchased from Cell Signaling Technology [Beverly, MA, USA]. Anti-IκBα monoclonal antibody [clone 6A920] was obtained from Caymen [Ann Arbor, MI]. Rabbit polyclonal anti-human SDF-1 [CXCL12] antibody was obtained from Novus Biologicals [Littleton, CO]. Rabbit polyclonal anti-CXCR4 antibody was obtained from Abcam [Cambridge, UK]. Rabbit monoclonal FAK Antibody [EP695Y] was purchased from Novus Biologicals [Littleton, CO]. Monoclonal Mouse IgG1 anti human αVβ3 [Clone 23C6] was obtained from R&D Systems [Minneapolis, MN]. Anti-human integrin α5β1 monoclonal antibody [clone JBS5] was obtained from Bioscience Research Reagents [formerly Chemicon] [Temecula, CA]. Anti-EPO monoclonal antibody was purchased from R&D Systems [Minneapolis, MN]. Polyclonal rabbit anti-Endothelin-1 [ET-1] antibody was purchased from Abbiotec [San Diego, CA]. Monoclonal mouse anti-MMP-9 antibody was purchased from Neuromab [Davis, CA]. Rabbit anti-human β-actin monoclonal antibody was purchased from OriGene Technologies [Rockville, MD]. Rabbit anti-human IgG was purchased from Abcam [Cambridge, MA] and was used as an isotype control antibody for Western Blot and immunohistochemistry studies.

**Figure 1:** YC-1 Exhibits Anti-Proliferative and Anti-Chemotactic Activities Under a Hypoxia-Independent Microenvironment in hRMVECs. **A. Chemical structure of YC-1. B. Cell Proliferation Assay.** YC-1 Inhibited VEGF-stimulated proliferation of hRMVECs that were grown for 48 hours. Treatments with SN50 or YC-1 for 48 hours suppressed VEGF-induced ECs growth. Whereas treatments with DMSO or SN50M had no impact on cell proliferation. Evaluation of DNA contents reflected the proliferative vitality rates in different groups. Values are presented as mean ± SEM obtained from triplicate experiments [*P<0.05; **P<0.01; ***P<0.001]. **C. YC-1 Inhibits hRMVECs Chemotaxis.** VEGF_165_ caused a significant increase in hRMVECs chemotaxis [***P<0.001] as compared to cells that were cultured in medium only. Treatment with YC-1 inhibits VEGF-induced cell migration. The inhibitory effects of SN50 as compared to SN50M exhibited the specificity of NFκB-mediated increase in chemotaxis induced by VEGF. The lack of VEGF presence in the control medium has significantly suppressed the hRMVECs migratory ability. Means ± SEM obtained from 6 wells/treatment of 4 independent experiments [*P<0.05; **P<0.01; ***P<0.001 vs. DMSO-treated cells].

### Tissue Culture

Human retinal microvascular endothelial cells [hRMVECs], attachment factor, complete growth medium were purchased from Cell Systems [Kirkland, WA]. Cells were cultured in 75-cm^2^ tissue culture flasks coated with attachment factor maintained in CS-C medium containing 10% FBS and CS-C growth factor at 1X in humidified conditions [5% CO_2_] at 37°C.

### Assessments of Cell Proliferation

hRMVECs [40,000 cells/well] were grown in a 96-well plate and cultured in 150 ml of CS-C medium supplemented with 10% FBS, placed in a CO_2_ incubator at 37°C and allowed to adhere overnight. Fresh medium was added and the cells were cultured for 48 hours at 37°C in CS-C medium and under one of the following conditions; VEGF-stimulated [30 ng/ml], VEGF-stimulated/DMSO-treated [0.2%], VEGF-stimulated/SN50M-treated [20 µM], VEGF-stimulated/SN50-treated [100 µM], or VEGF-stimulated/YC-1-treated [100 µM]. In each of these experiments, the cells were lysed in 0.1% sodium dodecyl sulfate [SDS]; DNA content was measured by means of Hoechst-33258 dye and a fluorometer [model TKO-100; Hoefer Scientific Instruments, San Francisco, CA]. It has been shown that total cellular DNA content measured in this manner correlates closely with actual cell number, as determined by hemocytometer counting of trypsinized retinal ECs.

### Chemoinvasion Assay

The invasiveness of hRMVECs was examined in vitro using a QCM™ 24-Transwell fluorimetric cell migration assay with polycarbonate filter inserts with 8.0-µm-sized pores. Briefly, the lower side of the filter was coated with gelatin [10 µl, 1 mg/ml], and the upper side was coated with Matrigel [10 µl, 3 mg/ml]. HRMVECs were grown to confluence in CS-C medium. To ensure precise results, hRMVECs cells were starved for 24 hours prior to the assay serum-free CS medium. HRMVECs cells [1×10^5^ cells] were suspended in 200 µl of serum-free CS-C medium with 0.1% bovine serum albumin and loaded into the upper chamber of a transwell. YC-1 [100 µM], or DMSO [0.2%], or SN50 [20 µM], or SN50M [20 µM] were added 1 hour before the assay and remained in the culture throughout the experiment. VEGF was diluted to 30 ng/ml in 0.6 ml of M199/0.1% bovine serum albumin and added to the lower wells of the chamber. Other lower wells were left with medium only. The chambers were incubated for 24 hour at 37°C in an atmosphere of 95% air and 5% CO_2_. The migrated cells were fixed with cold 70% methanol for 15 minutes and stained with the CyQuant Cell Stain Solution [Chemicon, CA]. The dye mixture was transferred to a 96-well microtiter plate suitable for measurement. Cell migration was identified by fluorescence plate reader using 480/520 nm filter.

### In vitro Angiogenesis Assay

The assay was conducted according to the manufacturer’s instruction [Chemicon, Temecula, CA] with modifications. Matrigel [10 mg/mL] was added to a 48-well plate and allowed to polymerize for 1 hour at 37°C. HRMVECs [6×10^4^] were seeded onto the surface of the matrigel and cultured in CS-C medium, under one of the following conditions; VEGF-stimulated [30 ng/ml], VEGF-stimulated/DMSO-treated [0.2%], VEGF-stimulated/SN50M-treated [20 µM], VEGF-stimulated/SN50-treated [100 µM], or VEGF-stimulated/YC-1-treated [100 µM]. DMSO, YC-1, SN50, SN50M, were added 30 minutes prior to the incubation. Tube-like structure formation was examined 24 hours after treatment. The enclosed networks of complete tubes from four randomly chosen fields/well at a magnification of X10 objective were photographed using inverted bright field microscopy [Zeiss Axiovert 135, Thornwood, NY]. Cells were labeled by adding 50 ml/well of Calcein AM [8 mg/ml]. Images were acquired using fluorescence microscopy [Zeiss Axiovert] and a digital camera [AxioCam, NY]. A mean of the total tube length at the four different fields was determined by Axiovision® 3.1 software and measured according to the branching points between two ECs. The images were printed at a constant magnification, and the length of the tubes formed was measured using the Axiovision imaging software [Zeiss], followed by calculation of the total relative length of the tube-like structures formed as percentage to the control. The inhibition percentage was calculated using the following formula: IR = [1–(tubes YC-1/tubes control)]×100%.

### Measurements of hRMVECs Lumen Formation

The assay was conducted according to the manufacturer’s instruction [Chemicon, Temecula, CA] with modifications. Matrigel [10 mg/ml] was added to a 48-well plate and allowed to polymerize for 1 h at 37°C. HRMVECs [6×10^4^] were suspended in 3D collagen gels and cultured in CS-C medium for 24 hours. The effects of exogenous addition of VEGF, DMSO, SN50M, SN50, and YC-1 on EC lumen formation over the time course of 24 hours were evaluated. Immunofluorescence still photography was performed using a fluorescence microscopy [Zeiss Axiovert] and a digital camera [AxioCam, NY]. After image acquisition, the values of immunofluorescence staining were analyzed and quantified using Metamorph™ imaging analysis software version 6.0 [Universal Imaging, Sunnyvale, CA]. EC Lumen areas per high power field were determined by tracing EC lumens using Metamorph software from acquired images.

### Evaluation of NFκB/p65 Transcription Factor Activity [ELISA]

ELISA assay was done after culturing the cells for 18 hours at 37°C in CS-C medium, under one of the following conditions; VEGF-stimulated [30 ng/ml], VEGF-stimulated/DMSO-treated [0.2%], VEGF-stimulated/SN50M-treated [20 µM], VEGF-stimulated/SN50-treated, or VEGF-stimulated/YC-1-treated [100 µM]. DMSO, YC-1, SN50, SN50M, were added 30 minutes prior to the incubation. Activation of the transcription factor NFκB was measured using a DNA-binding assay [Trans-AM™ NFκB/p65 Transcription Factor Assay Kit, Active Motif, Carlsbad, CA] according to manufacturer’s instructions. This is an ELISA-based method designed to specifically detect and quantify NFκB/p65 subunit activation, with high sensitivity and reproducibility. Nuclear protein extract was obtained using Nuclear Extract Kit [Active Motif] according to manufacturer’s instruction. Subsequently, a specific double stranded DNA sequence containing the NFκB response element was immobilized onto the bottom of the wells of the plate. Fifty [50 µg] of nuclear proteins were prepared, added to the wells, and incubated overnight at 4°C. NFκB binding specifically to the NFκB response element was detected by addition of specific primary antibody directly against NFκB/p65. A secondary antibody conjugated to HRP was added and incubated for 1 h at room temperature to provide a sensitive colorimetric readout at 450 nm.

### Subcellular Fractionation: Cytoplasmic and Nuclear Fractions

Adherent cells were scraped into ice-cold PBS harvested by centrifugation and washed once with ice-cold PBS. Cell-pellets were then lysed in hypotonic lysis buffer [5 mM HEPES, 1 mM MgCl2, 0.2 mM EDTA, 0.5 M NaCl, 25% glycerol, pH 7.0]. After incubation on ice for 10 minutes, lysates were centrifuged [13,000 *g*, for 5 minutes, at 4°C] to remove nuclei and cell debris. The cleared lysates were then removed to fresh tubes, frozen and stored at –20°C for subsequent estimation of protein concentration and use in Western blotting. The nuclei pellets were resuspended in hypertonic extraction buffer [10 mM HEPES, 1.5 mM MgCl2, 10 mM KCl, pH 7.9] for 1–2 hours at 4°C under agitation. After centrifugation [13,000 *g* for 10 minutes at 4°C], supernatants containing the nuclear protein were removed to fresh tubes and stored at –70°C. Protein concentrations were assessed by reaction with Bradford reagent [0.1% Coomassie blue G, 5% methanol, orthophosphoric acid].

### Western Blot

To determine the effects of YC-1 on VEGF-dependent IκBα phosphorylaion and degradation, and p65 translocation; hRMVECs were seeded overnight in 6-well plates [2×10^6^/ml]. Subsequently, hRMVECs were cultured for 8 hours at 37°C in CS-C medium, under one of the following conditions; VEGF-stimulated [30 ng/ml], VEGF-stimulated/DMSO-treated [0.2%], VEGF-stimulated/SN50M-treated [20 µM], VEGF-stimulated/SN50-treated, or VEGF-stimulated/YC-1-treated [100 µM]. DMSO, YC-1, SN50, SN50M, were added 30 minutes prior to the incubation. Cytoplasmic and nuclear extracts were prepared as previously described in the “Subcellular Fractionation: Cytoplasmic and Nuclear Fractions” section. Nuclear fraction was collected to examine the effects of YC-1 on nuclear translocation of p65. The protein concentration was determined using the Bradford assay [Bio-Rad] with BSA as a standard. Equal amount of cytoplasmic protein [30 mg] was resolved on 10% SDS-PAGE gel. Separated proteins were transferred to a nitrocellulose membrane [Roche, USA]. To avoid unspecific binding, the membranes were incubated in TBS containing 5% skim milk and 0.1% Tween 20 for 1 h at room temperature, and then immunoblotted with specific antibodies against; IκBα [1∶1000], phosphorylated IκBα [1∶1000], and β-actin [1∶1000]. To determine the effect of YC-1 on p65 translocation, 50 µg of nuclear protein were resolved on 10% SDS-PAGE, transferred and blotted with specific p65 antibody [1∶1000]. Negative control experiments consisted of omission of the primary antibody and utilizing a rabbit anti-human IgG [isotype control antibody] as a replacement. All the membranes were incubated overnight at 4°C. The membranes were washed, exposed to horseradish peroxidase-conjugated secondary antibodies for 1 h at room temperature, and finally the blots were detected by enhanced chemiluminescence reagent [Amersham Pharmacia Biotechnology, Little Chalfont] and analyzed using Quantity One software [BioRad, USA].

In another set of experiments; we investigated the influence of YC-1 on the protein expression levels of other molecules [SDF-1, CXCR4, FAK, αVβ3, α5β1, EPO, ET-1, and MMP-9]. Briefly, hRMVECs were seeded overnight in 6-well plates [2×10^6^/ml]. Subsequently, hRMVECs were treated with YC-1 [100 µM], or DMSO [0.2% *v/v*], SN50 [20 µM], or SN50M [20 µM] and then stimulated with 30 ng/mL VEGF for 48 hours at 37°C. Reactions were terminated by addition of lysis buffer [Cell Signaling, Beverly, MA]. Protein content of the cell lysates was determined according to the Bradford method [Bio-Rad, Hercules, CA]. Aliquots [40 µg] of whole-cell lysates were separated on 7.5% SDS-PAGE, and electro-transferred onto polyvinylidene membranes [Amersham Pharmacia Biotech, Little Chalfont]. After blocking with 5% nonfat dry milk in TBS-T, the blots were incubated overnight with anti-[SDF-1, CXCR4, FAK, αVβ3, α5β1, EPO, ET-1, MMP-9, and β-actin] antibodies. Negative control experiments consisted of omission of the primary antibody and utilizing a rabbit anti-human IgG [isotype control antibody] as a replacement. Then blots were washed 3×10 minutes washes in PBS/tween and subsequently incubated with peroxidase-conjugated anti-mouse IgG secondary antibody at 1∶3000. The signals were obtained by enhanced chemiluminescence [Amersham Biosciences], and visualized by exposure to X-ray film. Upon completion of chemiluminescence, equal lane loading was checked by Ponceau S Solution [Sigma, St. Louis, MO]. X-ray films were scanned with a computer-assisted densitometer [model G-710; Bio-Rad] to quantify band optical density [Quantity One software; Bio-Rad].

### Immunocytochemistry: Immunolocalization of NFκB/p65

The effect of YC-1 on the nuclear translocation of p65 was examined by immunocytochemistry. Briefly, hRMVECs [10^5^ cells/well] were grown on 8-well chamber slides and cultured for 8 hours at 37°C in CS-C medium and under one of the following conditions; VEGF-stimulated [30 ng/ml], VEGF-stimulated/DMSO-treated [0.2%], VEGF-stimulated/SN50M-treated [20 µM], VEGF-stimulated/SN50-treated, or VEGF-stimulated/YC-1-treated [100 µM]. DMSO, YC-1, SN50, SN50M, were added 30 minutes prior to the incubation. The cells were fixed with 3.7% paraformaldehyde and permeabilized with 0.2% Triton™ X-100 in PBS. The cells were incubated for 2 hours with anti-NFκB/p65 antibody. Negative control experiments consisted of omission of the primary antibody and utilizing a rabbit anti-human IgG [isotype control antibody] as a replacement. Cells were then incubated with HRP-conjugate working solution, followed by the addition of the Tyramid solution [TSA Kit#4] at 1∶100 dilutions [Molecular Probes, Carlsbad, CA]. Digitized images were acquired utilizing AxioVision software [Zeiss Axiovert 135 and AxioCam]. Intensity values of immunofluorescence staining of NFκB/p65 in cells was analyzed and quantified using Metamorph™ imaging analysis software version 6.0 [Universal Imaging, Sunnyvale, CA]. The staining intensity in our series ranged from a weak blush to moderate or strong. The amount of cells staining with the antibody was further categorized as focal [<10%], patchy [10%–50%], and diffuse [>50%]. For semiquantitative analysis, focal and/or weak staining was considered equivocal staining, and patchy or diffuse staining was subcategorized as either moderate or strong.

### ELISA: Measurements of the Nuclear Translocation of NFkB/p65

Cells [10^6^ cells/well] were cultured for 8 hours at 37°C in CS-C medium and under one of the following conditions; VEGF-stimulated [30 ng/ml], VEGF-stimulated/DMSO-treated [0.2%], VEGF-stimulated/SN50M-treated [20 µM], VEGF-stimulated/SN50-treated, or VEGF-stimulated/YC-1-treated [100 µM]. DMSO, YC-1, SN50, SN50M, were added 30 minutes prior to the incubation. The relative increase of NFκB/p65 translocation into the nucleus was measured using an ELISA according to the manufacturer’s protocol [IMGENEX, San Diego, CA]. In brief, the cells were centrifuged at 400 g for 1 minute and washed with cold PBS. The cells were lyzed by 400 µl of hypotonic buffer and 30 µl of 10% NP-40 was added. The mixture was centrifuged at 18000 g for 30 s. The supernatant was used as cytoplasmic extract. To the pellet was added 220 µl of nuclear extraction buffer and centrifuged at 18000 g for 1 minute. The supernatant was used as nuclear extract. The anti-p65 antibody coated plate captured nuclear or cytoplasmic free p65 of samples [0.5–1 mg/ml of protein] and the amount of bound p65 was detected by adding a secondary antibody followed by alkaline phosphatase-conjugated secondary antibody. The absorbance value for each well was determined at 405 nm by a microplate reader [Bio-Rad]. The relative ratio of nuclear to cytoplasmic p65 was calculated from the absorbance value of nucleus divided by that of cytoplasm.

### Quantitative RT-PCR by Molecular Beacon Assays

The mRNA levels for all genes [*NFκB/p65, SDF-1, CXCR4, FAK, αV, α5, β3, β1, EPO, ET-1, and MMP-9*] were quantified by Real time RT-PCR using specific primers. Gene-specific molecular beacons and primers were designed to encompass the genes of interest, with beacon’s annealing site to overlap with the exon-exon junctions for additional specificity [Beacon Designer 6.0, Premier Biosoft International, Palo Alto, CA, USA]. Threshold cycle [Ct] values for the different samples were utilized for the calculation of gene expression fold change using the formula 2 to the minus power of delta delta ct. Fold changes in the [*NFκB/p65, SDF-1, CXCR4, FAK, αV, α5, β3, β1, EPO, ET-1, MMP-9]* genes relative to the *β-actin* endogenous control gene were determined by the following equation: fold change = 2^–Δ [Δ*C*^_T_^]^, where change in threshold cycle [Δ*C*_T_] = *C*_T_ [*gene of interest*] – *C*_T_ [*β-actin*] and Δ [Δ*C*_T_] = Δ*C*_T_ [treated] – Δ*C*_T_ [untreated].

### Statistical Analysis

Data are given as means ± S.E.M. All experiments were repeated at least three times independently. Statistical analysis between two groups was performed using Student’s *t*-test. One-way ANOVA, combined with Tukey’s multiple-comparison test, was used to evaluate the statistical significance of differences between three or more groups. Statistical significance was defined as *P<0.05; **P<0.01; ***P<0.001.

## Results

### YC-1 Specifically Inhibits VEGF-stimulated Proliferation of hRMVECs

To determine whether YC-1 [Fig. 1A] could suppress VEGF-induced cell proliferation, hRMVECs were stimulated with VEGF [30 ng/ml] for 48 hours and DNA content was evaluated. VEGF_165_ induced a significant increase in hRMVECs proliferation, by 70.8% ±0.1% [***P<0.001], as compared to cells that were cultured in the absence of VEGF [medium only] [Fig. 1B]. However, the proliferation rate was reduced to 80% ±0.02 [***P<0.001] in the presence of 100 uM YC-1, as compared to DMSO-treated cells. Treatment with SN50 [20 uM] for 48 hours suppressed VEGF-induced ECs growth by 86.2% ±0.3 [***P<0.001] as compared to mutated control peptide, SN50M [20 µM]. The IC_50_ value for the antiproliferative effects of YC-1 in the presence of VEGF was 55.30±0.1 µM. Dye-exclusion assay revealed that there were no significant differences observed in cell viabilities between YC-1-treated cells, as compared to DMSO-treated controls [data not shown].

### YC-1 Inhibits hRMVECs Chemotaxis

VEGF_165_ caused a significant increase in hRMVECs chemotaxis [***P<0.001] [Fig. 1C]. This increase was inhibited by 4.65 folds in the presence of 100 uM YC-1 [***P<0.001], as compared to DMSO-treated cells. To determine whether NFκB induced the ECs activation and chemotaxis; NFκB peptide inhibitor, SN50 [20 µM] was added. Our results indicated that SN50 caused the inhibition of VEGF-induced chemotaxis by 7.50 folds, as compared to the mutated control peptide, SN50M [20 µM] treated cells. Under such conditions, no inhibition was observed indicating the specificity of NFκB-mediated increase in chemotaxis induced by VEGF. Cells that were incubated in medium only, exhibited an 815 folds decrease in their migratory ability, as compared to the VEGF-treated cells [***P<0.001].

### Anti-angiogenic Effects of YC-1 on VEGF-induced Tube Formation

HRMVECs cultured on the surface of three-dimensional type I collagen gel have a cobblestone-like appearance when cultured in the absence of VEGF [Fig. 2A]. Stimulation of hRMVECs with VEGF_165_ [30 ng/ml] induced the formation of three-dimensional capillary-like tubular structures within 24 hours [Fig. 2B]. Furthermore, VEGF stimulation increased the elongation of these structures, and augmented the numbers of their tube multicentric junctions. Treatment of hRMVECs with SN50M or DMSO didn’t have any influence on the growth or the integrity of these tube-like structures [Fig. 2C and 2D]. The angiogenic ability of hRMVECs to spontaneously form branching and thick anastomosing capillaries *in vitro* was severely abrogated by either SN50 [20 uM] [Fig. 2E] or YC-1 [100 uM] [Fig. 2F], as compared to their respective controls; SN50M- or DMSO-treated cells, respectively. Tubular morphogenesis, an indicator of NV, was significantly abrogated at 24 hours after SN50- or YC-1-treatments. SN50 and YC-1 blocked VEGF-promoted angiogenesis, as evidenced by the significant shortening of the capillary tubules and the presence of isolated cell clumps with few sprouting capillaries. The mean tube lengths were 101±2 um and 160±21 um in the presence of SN50 and YC-1, respectively. This represented a significant decrease of 81% ±0.03 and 77% ±0.02 in tube length in the presence of SN50 and YC-1, respectively [***P<0.001], as compared to their respective controls; SN50M- and DMSO-treated cells, respectively [Fig. 3A]. SN50 and YC-1 treatments significantly [**P<0.01] decreased the number of lumen formed in these ECs by 76% ±0.03 and 70% ±0.1, respectively [Fig. 3B], as compared to their respective controls; SN50M- and DMSO-treated cells, respectively.

**Figure 2:** YC-1 Displays Anti-Angiogenic Properties via the Inhibition of VEGF-Stimulated Tube Formation of hRMVECs. Representative micrographs exhibit the presence of cobblestone-like appearance when cells are grown in the absence of VEGF [A]. In the control groups [B, C, and D]; exposure of hRMVECs to VEGF_165_ [30 ng/ml] within 24 hours caused a rapid alignement of cells with one another to form tube-like structures. VEGF stimulation caused an increase in the elongation of the tube-like structures and the numbers of their tube multicentric junctions. Treatment with SN50 [E] or YC-1 [F] or caused a severe abrogation to the tube formation. Scale bars 75 mm.

**Figure 3:** Assessments of the Inhibitory Effects of YC-1 on hRMVECs. A. Quantitative Assessments of the Inhibitory Effects of YC-1 on Tube Formation. The capillary tubules were significantly shortened when treated with YC-1 or SN50, as compared to their respective controls; DMSO or SN50M, respectively. Data represent means ± SEM from three independent experiments with 3 replications in each experiment [*P<0.05; **P<0.01; ***P<0.001, as compared with the DMSO-treated controls by Student’s two-tailed t-test]. B. Quantitative Assessments of the Inhibitory Effects of YC-1 on Lumen Formation. The EC lumenal area were quantitatively measured over 24 hours by tracing EC lumenal areas using the Metamorph software program in order to systemically analyze EC lumen formation. The effects of addition of VEGF, DMSO, SN50M, SN50, and YC-1 on EC lumen formation over the time course of 24 hours, with the bar graph highlighting EC lumens per high power field [HPF] at 24 hour time point. SN50 and YC-1 treatments significantly [***P<0.001] decreased the number of lumen formed in hRMVECs as compared to their respective controls, SN50M and DMSO, respectively. Graph showing the mean number of EC lumens per high power field [HPF] ± S.D. [n = 3]. ***P<0.001; **P<0.01, as compared with controls.

### YC-1 Inhibits VEGF-induced NFκB Activation

In order to determine that VEGF effects on hRMVECs were mediated via the increase in the level of NFκB binding activity, we measured the NFκB/p65 activity by ELISA in hRMVECs, as compared to cells cultured in medium only [Fig. 4A]. VEGF induced a significant [***P<0.001] [98.3% ±0.01] upregulation in NFκB/p65 binding activity, as compared to cells that were incubated in medium only [no VEGF]. Treatment of cells with SN50 or YC-1 resulted in a significant [***P<0.001] attenuation of the VEGF-induced activation of NFκB binding activity. The extent of NFκB/p65 inhibition with SN50 or YC-1 was found to be 85% ±0.01, and 67% ±0.4, respectively, as compared to their respective controls; SN50M- and DMSO-treated cells, respectively [Fig. 4A]. Taken together, these data demonstrate that VEGF-stimulated effects are mediated via the activation of NFκB pathway, and YC-1 significantly inhibits such activity.

**Figure 4:** YC-1 Impairs VEGF-Induced NFκB Activation by Inhibiting IκBα Phosphorylation in VEGF-Treated Cells. **A. The Influence of YC-1 on VEGF-Induced NFκB Transcriptional Activity.**The graph illustrates the suppression of NFκB Activation by YC-1 in hRMVECs. ELISA assay was done after 18 hours of incubation with YC-1. Columns represent the means derived from three individual experiments. [*P<0.05; **P<0.01; ***P<0.001, as compared with controls. **B. Inhibition of IκBα Phosphorylation and Accumulation of IκBα by YC-1.** Cells were incubated in the absence or presence of 100 µl YC-1 for 8 hours. Cell extracts were then subjected to Western blotting using IκBα and p- IκBα antibodies. The blots exhibit the inhibitory influence of SN50 and YC-1 on the expression of the phosphorylated form of IκBα. **C. The Effects of YC-1 on Intranuclear Expression of NFκB/p65.** Cells were treated with one of the following conditions; DMSO, SN50M, SN50, or YC-1 in the presence or absence of VEGF for 8 hours. Nuclear extracts were prepared and assayed for NFκB/p65 by Western-blot as described in materials and methods. Both SN50 and YC-1 specifically inhibited the intranuclear expression of NFκB/p65 in cell preparations.

### Inhibition of IκBα Phosphorylation and the Accumulation of IκBα in YC-1-treated Cells

In order to determine; 1) whether VEGF influence on hRMVECs was mediated via NFκB pathway; and 2) whether the inhibition of NFκB activation by YC-1 was due to decreased degradation of IκBα, we examined IκBα degradation in response to VEGF stimulation. Because the degradation of IκBα normally requires the inhibitor to be phosphorylated, it was of interest to examine the extent of IκBα phosphorylation in SN50- and YC-1-treated cells, as compared to their respective controls; SN50M- and DMSO-treated cells. Western blotting for IκBα was done as an index of total inhibitor expression levels. Our data demonstrate that VEGF treatment promoted NFκB/p65 activation via upregulating the phosphorylation status of IκBα, which peaked at 8 hours following exposure to VEGF_165_; in addition, it increased its intrinsic hydrolysis activity [Fig. 4B]. Furthermore, our data reveal that blockade of IκBα phosphorylation with the specific NFκB inhibitor, SN50 [20 µM], significantly [***P<0.001] attenuated VEGF-stimulated IκBα phosphorylation, as compared to its respective control SN50M [Fig. 4B]. Likewise, the effects of VEGF on IkBα phosphorylation and degradation was significantly attenuated [***P<0.001] in the presence of YC-1 [100 µM] as compared to DMSO-treated cells [Fig. 4B]. Taken together, SN50 and YC-1 induced significant downregulations in the expression level of the phosphorylated form of IκBα [p- IκBα], while it induced significant upregulations in the levels of total IκBα expression levels, as compared to their respective controls; SN50M- and DMSO-treated cells, respectively [Fig. 4B]. These results are indicative that YC-1 induced the downregulation of the NFκB activity via; 1) blocking the degradation of IκBα; and 2) promoting the dephosphorylation and the accumulation of IκBα.

### YC-1 Impairs VEGF-induced Nuclear Translocation of NFκB/p65 Subunit

The effects of YC-1 on NFκB signaling were further explored by examining the nuclear translocation of the NFκB/p65 subunit in controls versus treated hRMVECs preparations. Our Western blot studies have indicated that SN50- and YC-1-treatments inhibited the nuclear translocation of NFκB/p65 protein, as compared to their respective controls; SN50M- and DMSO-treated cells [Fig. 4C].

In a different set of studies, our immunocytochemistry data have revealed that cells that were cultured in medium only exhibited the lack of p65 cytoplasmic and/or nuclear staining [Fig. 5A]. Whereas the cells that were stimulated with VEGF exhibited a significant increase [***P<0.001] in the signal intensity levels of dissociated nuclear p65, which was increased by 83.5 folds following VEGF treatment [Fig. 5B], as compared to cells that were cultured in medium only, which indicate that VEGF activates the canonical NFκB pathway. Cells that were stimulated with VEGF only, and/or treated with SN50M or DMSO; exhibited high levels of NFκB/p65 immunoreactivity, which was preferentially localized in the nuclei of the cells. In addition, there was a positive strong staining signal of NFκB/p65 deposited over the cytoplasms of the cells of these groups [Fig. 5B and 5C]. No NFκB/p65 staining was observed in experiments in which the primary antibody was omitted [data not shown]. Treatment of cells with SN50 or YC-1 had significantly abolished the VEGF-induced nuclear shuttling mechanism of p65 subunit, and ultimately blocked 88% and 82% of the VEGF-induced increase in NFκB/p65 levels, respectively, as compared their respective controls; SN50M-treated cells or DMSO-treated cells, respectively [Fig. 5C and 5D versus Fig. 5E and 5F]. Hence in the SN50 or YC-1-treated groups; the nuclear expression was virtually eliminated, yet few cells displayed the presence of cytoplasmic localization but then with equivocal “moderate or weak” staining intensity, in addition, a few stained regions were still detected in the nuclei. We demonstrate that VEGF-induced nuclear translocation of NFκB/p65 was severely abrogated in the presence of YC-1. This is in parallel with our Western blot data, which indicated a significant downregulation in the nuclear p65 levels in the SN50- and YC-1-treated groups. Taken together, these data indicate that YC-1 impairs VEGF-induced NFκB/p65 nuclear translocation.

**Figure 5:** YC-1 Impairs VEGF-Induced Nuclear Translocation of NFκB. A–F. Immunofluorescence Analysis. hRMVECs were incubated for 8 hours under various conditions and were subsequently fixed for immunocytochemistry. The staining intensity and the subcellular localization of NFκB/p65 were determined by immunofluorescence microscopy using anti-NFκB/p65 antibody. Photomicrographs, which exhibit intense nuclear and/or cytoplasm staining was considered a positive signal. Cells that were stimulated with VEGF alone (B), or incubated with either VEGF/SN50M (C) or VEGF/DMSO (D); exhibited high levels of NFκB/p65 immunoreactivity, which was preferentially localized in the nuclei of the cells. In addition, there was a positive intense staining signal of NFκB/p65 deposited over the cytoplasms and nuclei of the cells of these groups. Treatment of cells with SN50 [20 uM] or YC-1 [100 uM] resulted in a significant and almost complete inhibition of NFκB/p65 nuclear translocation. Images are representatives of three independent experiments. Scale bars, 200 mm.

In another series of experiments, cells were treated with either; YC-1 [20 µM], or DMSO [0.2%], or SN50 [20 µM], or SN50M [20 µM] in the presence or absence of VEGF [30 ng/ml], and later cells were analyzed by two different types of ELISA assays. The first ELISA assay detected the nuclear translocation of p65 [Fig. 6A], while the second assay was utilized to further quantify the nuclear/cytoplasmic ratio of p65 [Fig. 6B]. To conduct both assay, nuclear protein extracts were prepared from hRMVECs after exposure to VEGF_165_ [30 ng/ml]. Our results indicated that VEGF induced a significant [***P<0.001] increase 94.6% ±0.04 in NFκB/p65 nuclear translocation, as compared to cells cultured in medium only. Furthermore, treatment of cells with SN50 or YC-1 significantly [***P<0.001] reduced the nuclear NFκB/p65 translocation by 83.5% ±0.2 and 77% ±0.03, as compared to their respective controls; SN50M-and DMSO-treated cells, respectively.

**Figure 6:** YC-1 Induced Specific Alterations in the Cytoplasmic-Nuclear Shuttling of NFκB/p65. A. ELISA Assay Analysis: YC-1 Inhibits Nuclear Translocation of NFκB/p65. The relative nuclear translocation of NFκB/p65 in hRMVECs was measured by ELISA. ELISA was performed as described in Materials and methods. NFκB/p65 translocation to the nucleus was inhibited in YC-1- and SN50-treated cells. Data are expressed as Mean ± SD of triplicate cultures from at least three independent experiments. **B. The Relative Ratio of Nuclear to Cytoplasmic p65 in the Cells Treated with YC-1.** Data represent the mean ± SD of three [3] independent experiments. Statistical analysis was performed [*P<0.05; **P<0.01; ***P<0.001, as compared with the DMSO-treated cells by Student’s two-tailed t-test].

Our second ELISA assay has indicated that treatment of cells with SN50 or YC-1 resulted in a significant [***P<0.001] reduction in the p65 nuclear/cytoplasmic ratio, as compared to their respective controls; SN50M-treated and DMSO-treated cells, respectively [Fig. 6B]. These data are indicative that YC-1 inhibited nuclear translocation of NFκB/p65 subunit followed suppression of NFκB/p65 activity.

### YC-1 Downregulates the Pro-angiogenic Gene Expression Profile in VEGF-stimulated hRMVECs

We have utilized quantitative real time RT-PCR to elucidate the molecular mechanisms involved in the regulation of VEGF-induced NFκB-dependent retinal neovasculogenesis. The mRNA expression levels of; *NFκB/p65, SDF-1, CXCR4, FAK, αV, α5, β3, β1, EPO, ET-1, and MMP-9* were evaluated. The data were normalized to β-actin mRNA expression level. Our results demonstrate that there were significant upregulations in the message levels of the above mentioned pro-angiogenic genes in the VEGF-stimulated cells, as compared to cells that were cultured in medium only [Fig. 7A–F] and [Fig. 8A–E]. Treatment of hRMVECs preparations with YC-1 [100 µl] significantly downregulated the mRNA expression levels of the above mentioned genes, as compared with DMSO-treated cells. However, their expression level remained slightly higher than that of the cells that were cultured in medium only. The effects of sham treatment [DMSO] on the gene expression patterns paralleled those seen in the VEGF-stimulated cells. The mRNA expression levels of; *NFκB/p65, SDF-1, CXCR4, FAK, αV, α5, β3, β1, EPO, ET-1, and MMP-9* were evaluated by using the primers that were summarized in [Fig. 9A].

**Figure 7:** YC-1 Inhibits the Expression of *NFκB/p65, SDF-1, CXCR4, αV, α5,* and *β1* in VEGF Stimulated Cells. A–F. Real Time RT-PCR Analysis. The mRNA levels for *NFκB/p65, SDF-1, CXCR4, FAK, αV, α5, β3, β1, EPO, ET-1, MMP-9,* was quantified by Real time RT-PCR. The mRNA levels of these genes were upregulated in the cells that were cultured in the presence of VEGF [30 ng/ml] and either treated with DMSO [0.2%], or SN50M [20 µM]. Whereas the cells that were cultured in medium only exhibited significant low mRNA levels. Treatment of VEGF-stimulated cells with SN50 [20 µM] or YC-1 [100 µM] resulted in a significant downregulation of the mRNA expression of the genes listed above, as compared to respective controls; SN50M and DMSO-treated cells, respectively. ANOVA was used for statistical analyses. Mean ± SEM of mRNA level normalized to β-actin were calculated, [***P<0.001 and **P<0.01, as compared to respective controls]. Data are representative of 3 independent experiments.

**Figure 8:** YC-1 Inhibits the Expression of Various Pro-Angiogenic Molecules in VEGF-Stimulated Cells. **A–E. Real Time RT-PCR Analysis.** The mRNA levels for *β3, FAK, EPO, ET-1, and MMP-9,* was quantified by Real time RT-PCR. The expression level was upregulated in the cells that were cultured in the presence of VEGF and either treated with DMSO or SN50M. Treatment with SN50 or YC-1 resulted in a significant downregulation of the mRNA expression, as compared to their respective controls; SN50M and DMSO-treated cells, respectively. ANOVA was used for statistical analyses. Mean ± SEM of mRNA level normalized to β-actin were calculated, [***P<0.001 and **P<0.01, as compared to respective controls]. Data are representative of 3 independent experiments.

**Figure 9:** YC-1 Inhibits the Protein Expression of Various Pro-Angiogenic Molecules in VEGF-Stimulated Cells. **A. Sequence for the Primer Sets Used for the Quantitative Real-Time PCR Analysis.** **B. Western Blot Analysis.** Protein expression levels were significantly elevated in the cells that were treated with SN50M or DMSO in the presence of VEGF [30 ng/ml]. In VEGF-stimulated/SN50-treated [20 µM], and VEGF stimulated/YC-1 treated [100 µM] cells, the protein expression levels were significantly decreased, as compared with SN50M and DMSO-treated cells. Statistical significance was determined by ANOVA [**p<0.01]. Data are representative of 3 independent experiments.

#### YC-1 inhibits the pro-angiogenic proteins expression in VEGF-stimulated hRMVECs

Western blot analysis demonstrated that cell exposure to VEGF induced a significant [***P<0.001] upregulation in the expression levels of SDF-1, CXCR4, FAK, αVβ3, α5β1, EPO, ET-1, and MMP-9, as compared to cells that were incubated in medium only [Fig. 9B]. Treatment with YC-1 [100 µM] significantly inhibited the expression of levels [***P<0.001] of these proteins as compared to DMSO-treated cells [Fig. 9B]. Since YC-1 treatment did not inhibit β-actin, this indicates that YC-1 influence on the expression of the above proteins was specific.

## Discussion

Hypoxia-induced expression of VEGF is a crucial mechanism that triggers an angiogenic response under physiological and pathological conditions. VEGF has been proposed to play an important role in the pathogenesis of diabetic vascular complications. Therefore, with the progress of DR; retinal ischemia and subsequent hypoxia may become a major determinant of VEGF. It has been suggested that there is a significant elevation of VEGF levels in ocular fluids obtained from patients with DR [20]. Conversely, neutralizing anti-VEGF antibodies in experimental animals have been implicated in the inhibition of VEGF signaling, the suppression of retinal NV [21], and the reversal of high glucose–induced vascular hyperpermeability [22]. Our current study demonstrates that VEGF treatment in hRMVECs promotes NFκB activation via; 1) upregulating the phosphorylation status of IκBα and increasing its intrinsic hydrolysis activity; 2) promoting the nuclear accumulation of p65; and 3) increasing the NFκB activity. Whereas YC-1 treatment induced the downregulation of the NFκB activation by preventing IκBα degradation, and hence inhibiting the nuclear translocation of NFκB/p65 subunit.

Previous studies have indicated that NFκB can regulate VEGF transcription [23]. Analyses of the VEGF promoter have not identified consensus and functional κB sites [24], and therefore, NFκB may regulate VEGF indirectly through other transcription factors. Our data suggest a pivotal role of NFκB activation in the development of diabetic microvascular angiopathy under a hypoxia-independent mechanism. The current study reveals that treatment of hRMVECs with VEGF enhances NFκB binding activity and invokes the expression of several pro-angiogenic factors [SDF-1, CXCR4, FAK, αVβ3, α5β1, EPO, ET-1, and MMP-9] via NFκB-dependent mechanism. This upregulation was attenuated by the NFκB inhibitor SN50 and by YC-1 suggesting a common effecter target for the peptide SN50 and the sGC activator, YC-1. Our observations exhibits that YC-1 exerted an inhibitory effect on several essential steps of retinal neovasculogenesis, including cell invasion and migration, through NFκB signaling pathway. These observations are in parallel with previous studies, which indicated that YC-1 abolished constitutive nuclear translocation and activation of NF-kappaB/p65 in PC-3 cells [25]. Furthermore, it has been demonstrated that in STZ-induced diabetes, there was a significant increase in HIF-2α in the retinas of the diabetic rats, which was independent of hypoxia [12]. Our observations underscore the complexity and diversity of such neovascular angiogenic response, specifically in the absence of hypoxia.

During this investigation we report for the first time the molecular nexus between VEGF and NFκB in relation to retinal neovasculogenesis in the absence of the hypoxic microenvironment, and investigated the possible pathological role, which may play in instigating retinal NV. Furthermore, we have now analyzed the effects of YC-1 on VEGF-induced stimulation of NFκB, which mediated a significant upregulation in the expression of various pro-angiogenic molecules and augmented retinal neovasculogenesis in hRMVECs. The use of YC-1, with its pleiotropic effects [26], [27] may be necessary to offset such compensatory angiogenic responses and maximize therapeutic outcomes. Although our data may suggest the potential therapeutic use of YC-1 in ocular diseases, it is imperative that a suitable *in vivo* model is utilized to demonstrate the full potential of sGC agonists in retinal vasculopathy.
